The article "Blue prescription: A pilot study of health benefits for oncological patients of a short program of activities involving the sea" was published in 2023. Journal: Heliyon.

# Blue prescription: A pilot study of health benefits for oncological patients of a short program of activities involving the sea

**DOI:** 10.1016/j.heliyon.2023.e17713

**Published:** 2023-07-05

**Authors:** Arnau Carreño, Eva Fontdecaba, Angel Izquierdo, Olga Enciso, Pepus Daunis-i-Estadella, Gloria Mateu-Figueras, Javier Palarea-Albaladejo, Mireia Gascon, Cristina Vendrell, Montserrat Lloveras, Joan San, Sílvia Gómez, Stefania Minuto, Josep Lloret

**Affiliations:** a Sea Health, Oceans and Human Health Chair, Institute of Aquatic Ecology, University of Girona, C/ Maria Aurèlia Capmany 69, 17003, Girona, Spain; b Medicina de Familia, CAP Castelló D’Empúries, Donostia-San Sebastian, Spain; c Institut Català D'Oncologia, Hospital de Girona Dr. Josep Trueta, Avinguda de França S/n, 17007, Girona, Spain; d Medicina de Familia, CAP Tossa de Mar, Corporació de Salut Del Maresme I La Selva, Girona, Spain; e Dept. of Computer Science, Applied Mathematics and Statistics, University of Girona, Girona, Spain; f Barcelona Institute for Global Health (ISGlobal), Barcelona Biomedical Research Park (PRBB) Doctor Aiguader, 88 08003, Barcelona, Spain; g Universitat Pompeu Fabra (UPF), Barcelona, Spain; h CIBER Epidemiología y Salud Pública (CIBERESP), Madrid, Spain; i Medicina de Familia, CAP Roses, Girona, Spain; j Medicina de Familia, CAP Montilivi (Girona), Girona, Spain; k Dep. Social Anthropology, Autonomous University of Barcelona, Building B-Campus UAB, 08193, Bellaterra, (Cerdanyola Del Vallès) Barcelona, Spain

## Abstract

Performing outdoor activities in blue spaces can help improve human health and mental well-being by reducing stress and promoting social relationships. The number of people surviving cancer has increased globally to experience this disease as a life-changing and chronic condition with physical and psychosocial symptoms that have negative impacts on their quality of life. While there has been a growth of programs in green spaces to meet the needs of cancer patients, such as follow-up post-treatment care, support groups and physical activity programs, very few studies have examined the effects of activities involving the sea for the health and well-being of oncology patients. This is the first study to evaluate whether different outdoor activities in blue spaces can benefit oncological patients' physical and mental health using smartwatches, sphygmomanometers and Profile of Mood States (POMS) questionnaires. We assessed changes in blood pressure, heart rate, sleep quality and mental health of 16 patients after twelve sessions of three different activities (walking, beach and snorkelling) and four sessions of a control activity. While no significant differences between activities were observed in terms of the data gathered by the smartwatches, a gradient of positive results for human mental health was observed towards exposure to a blue space, assessed through POMS questionnaires. Results show that exposure to blue spaces contributes to tension and anger reduction and improves the vigour mood state of oncology patients. No significant increases in patients' heart rate were recorded after the beach and snorkelling activities, with results similar to the control activity, suggesting that the contribution may be to participants’ relaxation.

The article "Blue prescription: A pilot study of health benefits for oncological patients of a short program of activities involving the sea" was published in 2023. Journal: Heliyon.

## 1 Introduction

Research on the effects of being in touch with or exercising in blue spaces has rapidly expanded over the past decade [19,20,26,32,82]. In the European Commission funded project BlueHealth (https://bluehealth2020.eu/), blue spaces are defined as “natural or manmade outdoor environments that prominently feature water and are accessible to humans either proximally (being in, on, or near water) or distally/virtually (being able to see, hear or otherwise sense water)” [28].

The findings for blue spaces converge with those for green spaces, concluding that regular contact with natural environments can enhance well-being and alleviate stress [4,14,23,25,53,65,73]. There is growing evidence showing that exposure to blue spaces has potential benefits for mental health, well-being and the promotion of physical activity [8,22,24,25,37,39,82], and a wide range of programs have been developed to engage people in water sports - or so called “blue gym” or “blue care” activities [5,15,84]. Recent studies within the framework of the EU funded project BlueHealth have confirmed these associations [55,77,83]. Indeed, other studies have shown that non-motorised leisure or sport activities at sea, such as swimming, scuba diving and kayaking, can also have positive health outcomes for the users (reviewed by Refs. [5,32,37]. For instance, in a recent study we showed that short-term exposure to scuba diving could have mental health benefits for the general population, especially among those taking regular medication to treat chronic illnesses [8]. Therefore, getting in touch with or practicing sport in blue spaces can be used not only to prevent disease, but also to promote good psychological health and help individuals with chronic health conditions to manage their rehabilitation, recovery or ongoing health states [32,37,82]. However, the evidence base for the health or well-being benefits of therapeutic interventions in blue spaces has been scarcely studied.

Cancer has a very strong psychological component, producing a wide range of long-term psychological symptoms that have an impact on patients’ quality of life, including fear of cancer recurrence, fatigue, sleep, sexuality disturbances, anxiety and pain [1,49,61]. Cancer survivors can experience ongoing symptoms following treatment, particularly psychosocial symptoms [70], which can have a negative impact on their participation in daily activities and their quality of life (Silver & Gilchrist, 2011; [70]. Due to economic and time constraints, it is increasingly challenging for hospital-based services to fulfill the requirements of cancer survivors in terms of providing follow-up post-treatment care and support to increase activity participation [47,52]. Among the people suffering from chronic illnesses, cancer patients are considered to benefit significantly from engaging in sports activities (see e.g. Refs. [43,44,78].

The article "Blue prescription: A pilot study of health benefits for oncological patients of a short program of activities involving the sea" was published in 2023. Journal: Heliyon.

However, very few studies have examined the effects of activities involving the sea on the health and well-being of oncology patients. In studies evaluating the effects of dragon boat racing on participants recovering from breast cancer, positive psychosocial impacts and improvements in self-reported body image, confidence and socialization, among other outcomes, were observed [42]; T. L. [43]; T [44,54,67,78]. And while swimming is being prescribed for breast cancer patients, given the positive effects on physical and mental recovery [57], there are no studies on how a regular program of swimming or snorkelling in open waters may benefit both the physical and mental health of individuals coping with cancer.

Therefore, based on this previous scientific evidence, we hypothesized that engagement in marine leisure activities, such as walking by the sea, swimming, and snorkelling in well-preserved coastal and marine blue spaces, can lead to significant improvements in physiological parameters (e.g. heart rate and blood pressure), increased quality of sleep, and enhanced mental health and well-being in oncological patients.

Consequently, the purpose of this study was to assess the potential positive health effects of engaging in marine leisure activities in well-preserved blue spaces on the coast and in the sea for individuals with a history of cancer. The specific aims of this research were to investigate whether activities such as seaside walking, swimming, and snorkelling can lead to i) improvements in physiological indicators, such as heart rate and blood pressure; ii) enhancement of sleep quality; and iii) promotion of mental health and well-being among oncological patients.

## 2 Materials and methods

### 2.1 Setting and study population

The present study used a mixed-method design, combining qualitative and quantitative data, and was conducted over two summer seasons (years 2020 and 2021), on weekday mornings and afternoons, in the towns of Roses and Tossa de Mar, Catalonia, Spain. Both are towns on the Costa Brava, an iconic landscape and seascape of the northeastern part of Catalonia, which hosts a high biodiversity of marine species, and is highly valued by tourism. The area is visited by tourists from all over the world and has abundant marine and land activities and businesses operated by various local stakeholders (e.g. kayaking, scuba diving, etc.) (Fig. 1).

The article "Blue prescription: A pilot study of health benefits for oncological patients of a short program of activities involving the sea" was published in 2023. Journal: Heliyon.

**Fig. 1:** Location of Roses and Tossa de Mar in the Mediterranean Sea.

Recruitment of participants was coordinated by the Oceans and Human Health Chair, the local medical centeres of Roses, Castelló d’Empúries and Tossa de Mar (CAPs), and the Catalan Institute of Oncology (ICO), with the help of a local oncological patients' association (Fundació Roses Contra el Càncer). Potential participants were approached either by the physicians from the local CAPs or by the local association in Roses. Those interested in taking part had a personal interview with the local physicians taking part in the study, in which the objectives and requirements were explained. The medical records of those who agreed to take part were reviewed by the physician in charge of the ICO territorial section of Girona to confirm their eligibility. Accepted participants had an informative meeting with the research team physicians and investigators in order to get to know each other, to explain in detail the objectives and methodology of the study and to agree on joining a mobile phone messaging group to schedule the activities and sessions.

The criteria for the participants to be included in the study were: i) aged between 18 and 70 years; ii) at least 6 months post-treatment and not more than 5 years post-diagnosis; iii) non-active tumour in remission phase; iv) not having developed a tumour in the respiratory tracts or in areas that are incompatible with practicing water sports; v) knowing how to swim. Therefore, the exclusion criteria for the potential participants were the following: i) having an active tumour; ii) having received treatment within the past six months; iii) having been diagnosed with cancer for more than five years; iv) having developed a tumour in the respiratory tracts or areas that are incompatible with water sports; and v) not knowing how to swim or having fear of swimming in the sea. The study was approved by the ethics and biosecurity committee of the University of Girona (CEBRUdG) (CEBRU0007-2020) and the Ethics Committee of the University Institute for Primary Health Care Research (IDIAP) Jordi Gol (20/124-P).

The article "Blue prescription: A pilot study of health benefits for oncological patients of a short program of activities involving the sea" was published in 2023. Journal: Heliyon.

Confidentiality and anonymity of data were guaranteed by EU Regulation 2016/679 of the European Parliament and the Council, of 27 April, on Data Protection (GDPR) and the national regulations governing the development, presentation and publication of the results of this study.

### 2.2 Study design

Recruited participants took part in different activities, including walking by the sea and bathing/swimming and snorkelling in the sea, together with a control activity, which consisted of resting in a quiet room. Each of these activities was carried out over four sessions that lasted for approximately half an hour each, for a total of 16 sessions to complete the full program. Participants were always accompanied and supervised by the researchers, physicians and, in the case of the snorkelling sessions, also diving instructors who provided support and assistance to solve any inconvenience arising during the activities (e.g. assistance when entering the sea, smartwatch configuration, resolution of doubts when answering the questionnaires, etc.). More specifically, the activities that the patients took part in were the following (Fig. 2): i) walking: participants completed a 30-min low-demanding walking itinerary along the seafront with sea views at all times; ii) bathing from the beach: participants were asked to relax or swim in the sea for 30 min, but without swimming goggles; iii) snorkelling: participants were provided with snorkel masks and a wetsuit if required, and were asked to swim and observe the ecosystem on their own, following a low-demanding pre-defined route and always accompanied by a member of the research team and a diving instructor; and iv) control sessions: participants were asked to sit and relax in a comfortable office without views for 30 min. In the control sessions, participants could not use any mobile devices, listen to music, read or talk to other people.

**Fig. 2:** Schematic representation of the experimental design of the study.

### 2.3 Individual characteristics and well-being and mood state

Five different questionnaires were distributed to the participants during the study, who were asked to respond to the content just before and after taking part in the respective activity sessions (approximately 1 h between questionnaires). Background questionnaires were only completed once and included information on individual characteristics, their physical activity and their health. Activity-related questionnaires, which included information on perception of health and daily physical activity, were distributed before the first and after the last sessions of each activity. Questionnaires before and after each session included information on the quality of sleep of the previous night, characteristics of the activity and mood state questionnaires (Table 1). More information on the content of the questionnaires is available in Appendix 1.

The article "Blue prescription: A pilot study of health benefits for oncological patients of a short program of activities involving the sea" was published in 2023. Journal: Heliyon.

**Table 1:** Frequencies of distribution of the questionnaires.

Type of questionnaires	Nomenclature		Frequency
**Personal data**	Background Questionnaire		One-time only, distributed in the 3rd control session
**Activity related** (Included information on perception of health and physical activity)	Prior cluster of activity questionnaire	Posterior cluster of activity questionnaire	Questionnaires distributed in the first session and the last session of each activity
**Session related** (Included information on the quality of sleep and characteristics of the activity)	Prior session questionnaire	Posterior session questionnaire	Daily questionnaires distributed before and after the session
**Mood state**	POMS questionnaire before the activity	POMS questionnaire after the activity	Daily questionnaires distributed before and after the activity

The Profile of Mood States (POMS) questionnaire was distributed before and after each session to assess the effect of the “blue spaces” activities on participants’ mental health. Originally developed by McNair, Loor and Droppleman in 1971 [74], this is a well-established, academically and clinically validated measure of psychological distress and mental well-being consisting of 65 mood state questions grouped into 6 categories. POMS questionnaires have also been used in similar studies assessing the contribution of medium-term exposure to blue and urban spaces to the mental health of participants undertaking walking routines lasting some days (Vert et al., 2019). For this study, we used the 29-item version established by Ref. [21]; which divides mood states into 5 mood categories, and explains 92.9% of the covariance of the original questionnaire: tension/anxiety (TA), depression (D), anger/hostility (AH), fatigue (F), and vigour (V). Responses for each item were rated on a five-point scale ranging from “Not at all” to “Very much”. The total score for POMS before and after the activity was calculated using the following formula: [(TA) + (D) + (AH) + (F) – (V)]. Following this formula, higher POMS scores indicated worse psychological distress. To avoid negative numbers when fitting the model, we added 100 to the POMS final score (before and after the activity) [2].

### 2.4 Arterial blood pressure and heart rate

Before and after each session for each activity, participants’ systolic and diastolic arterial blood pressure (SBP & DBP) and heart rate (HR)were registered with a sphygmomanometer (Omron model M3 Comfort HEM-7155-E). Three measures of the parameters (i) systolic blood pressure, (ii) diastolic blood pressure and (iii) heart rate were taken simultaneously for each participant 5 min before each session. Ten minutes after the sessions, and after responding to the psychological questionnaire, the same three measures were again taken.

The article "Blue prescription: A pilot study of health benefits for oncological patients of a short program of activities involving the sea" was published in 2023. Journal: Heliyon.

### 2.5 Physical health parameters and smartwatches

We used the Polar Vantage M multisport GPS watch with wrist-based heart rate monitoring to assess the following physical parameters related to health: HR, total amount of sleep, sleep interruptions, sleep efficiency (%), deep sleep amount (%), and rapid eye movement (REM) sleep (%). Each participant was given a smartwatch along with an explanation of how their devices operated, and how to charge, wear, synchronize them. They were told to wear the devices 24 h a day with the wrist HR monitoring function on active. They could wear it on the right or left wrist, but were not allowed to change the initially chosen wrist. After waking up and before going to sleep, participants also had to synchronize their devices with the mobile phone application PolarFlow to ensure that the database was continually updated database. Moreover, while not directly taking part in the study, participants were allowed to use their smartwatches for their daily routines and activities to encourage its use and adaptation. Participants were required to activate the function “training session” depending on the organized activity they were taking part in (“walking” for control and walking sessions; and “open water swimming” for the beach and snorkelling sessions) just before starting the session and after having completed the questionnaires and blood pressure and HR recording. Immediately after the session, and before responding to the questionnaires, this function was deactivated and the session characteristics were recorded in a database (position, elevation gain, steps, HR, etc.).

### 2.6 Heart rate

Following the methodology of [75,76]; various 10-min periods were established to evaluate HR changes during resting times. These time points were the following, in chronological order: 10 min before waking up; the day of doing the activity (BWU1); 10 min after waking up (Waking up); 10 min before doing the activity (Before); 10 min after doing the activity to recover the usual HR (After); 10 min after going to bed at night (Sleep); and 10 min before waking up, the day after doing the activity (BWU2).

### 2.7 Quality of sleep

Insomnia affects up to 50% of patients with cancer, but it is a symptom that has often been overlooked by the oncology community when compared with other symptoms such as pain and fatigue [51]. Insomnia and subsequent sleep disturbances can lead to fatigue and mood disturbances, and contribute to immunosuppression, which can have a profound impact on quality of life and may contribute to increased mortality and morbidity of the disease [51]. Studies state that low levels of activity improve the sleep quality of patients with insomnia, decreasing depression symptoms and increasing overall mood [30,72].

The article "Blue prescription: A pilot study of health benefits for oncological patients of a short program of activities involving the sea" was published in 2023. Journal: Heliyon.

In this regard, studies show that sleep need is inversely correlated to REM density. In fact, 89% of the variance of the trend of REM densities after different sleep deprivation is explained by the linear component [38]. Therefore, assessing light, deep and REM density patterns and total quantity of sleep may be a good indicator of the quality of sleep of the study population.

We compared the quality of sleep the night before doing the activity with the quality of sleep the night after doing each activity (control, walk, beach and snorkelling). Moreover, four random nights were assessed per participant to compare them with the control nights (both the nights before and after the control sessions).

The smartwatch model used in this study provided a score ranging between 1 and 100, given by an internal algorithm that takes a number of variables into account (e.g. percentage and quantity of light, deep and REM sleep periods, interruptions, and overall quantity of sleep). In addition, information about the length and percentage of different sleep stages was provided by the devices (e.g. Light, Deep, REM sleeps and interruptions). We used both the scores and the percentages of sleep stages provided by the smartwatches to assess the quality of sleep.

### 2.8 Sample size

Constrained by the difficulties in recruiting participants and the risk of dropout in the context of the individual's illness and the Covid-19 pandemic, this study aimed to collect meaningful information from a minimally representative sample of participants from the two towns. In total, 21 participants aged between 35 and 70 years old met the inclusion criteria and were recruited within one year, 12 in Roses (11 females and one male) and nine in Tossa de Mar (four females and fives males). Participants had been diagnosed with different types of cancer including breast, bladder, testicle and colon. This sample was regarded as sufficient to gain initial insight into the research question and achieve a better understanding of the experimental setting to inform future studies.

All the participants in Roses completed all the stages of the study, while only three female participants and one male participant did so in Tossa de Mar. The others were able to complete the control and walking by the sea sessions but were not able to take part in the beach and snorkelling sessions for different reasons, including difficulties combining the sessions with their work schedule and health issues. Participants who were unable to complete all the stages were discarded from the data analysis since the comparison of activities in a blue space was the main objective of the study. Therefore, while the final study population included in the statistical analysis was 16 participants, only 12 of them had complete and useable data recorded by their smartwatches.

The article "Blue prescription: A pilot study of health benefits for oncological patients of a short program of activities involving the sea" was published in 2023. Journal: Heliyon.

### 2.9 Data analysis

All data analysis and statistical modelling was conducted using the R system for statistical computing v4.1.1 [60]. Statistical significance was generally concluded at the usual 5% significance level (p < 0.05).

#### 2.9.1 Statistical modelling of POMS data

The effects on POMS scores of the different activities and differences between the scores were statistically tested by fitting Poisson generalised linear mixed models (GLMMs) with a logarithmic link function to the post-activity POMS scores, including the pre-activity POMS scores as an offset (in log-scale), the activity group as a fixed effect, and session and individual ID as random effects. This model accounted for the counting nature of the POMS data, the baseline levels, the grouping structure determined by session, and the dependency between repeated measures taken on the same individuals. Based on previous literature, the following variables of adjustment were also included in the model: age, having children under 16, home with access to an open space, previous night's sleep quality and feeling safe while doing the activity [8]. GLMM selection was conducted by the likelihood ratio testing, considering different structures of fixed and random effects. The session number appeared not to be relevant as a random effect and only individual ID within location was included in the final model as a random effect. Post hoc pair-wise tests of differences in mean between activity groups were conducted based on the predicted marginal means from the GLMM estimates. The corresponding p-values were adjusted for multiplicity using the Benjamini and Hochberg's method [3].

#### 2.9.2 Statistical modelling of SBP, DBP and HR data registered using a sphygmomanometer

Linear mixed models (LMMs) were fit by restricted maximum likelihood to post-activity SBP, DBP and HR variables, with pre-activity values included as offsets. Both post- and pre-activity variables were log-transformed to better accommodate model normality assumption. The activity group was entered as a fixed effect, while the session and individual ID within location were considered as random effects. Based on the previous literature, the models were adjusted for some potential confounding variables: age, gender, height, weight, medication and pre-week/post-week activity (low, medium, high levels).

The article "Blue prescription: A pilot study of health benefits for oncological patients of a short program of activities involving the sea" was published in 2023. Journal: Heliyon.

#### 2.9.3 Statistical modelling of heart rate registered using smartwatches

Data for this analysis were only obtained from the 12 participants from Roses. To make the HR measurements comparable between participants across the different activities, the values registered for each time lapse were standardized relative to those obtained at the same times of day in the control sessions as a baseline. To this effect, each individual HR was subtracted from their baseline mean HR and divided by the standard deviation of the baseline HR (all values in natural log-scale to better approach normality assumption). These standardized HR values were used to fit a linear mixed model including activity, time point of measurement, and the interaction between them as fixed effects, along with individual ID and session as random effects. To prevent excessive sensitivity of the statistical tests to small effects derived from the large number of raw data points (>25,000), the model took as input the mean of the standardized HR values over the 10-min observation periods as a summary for each individual at every time point, activity and session. Post hoc pair-wise tests of differences in mean between activity groups were conducted based on the predicted marginal means from the LMM estimates. The corresponding p-values were adjusted for multiplicity using the Benjamini-Hochberg's method.

#### 2.9.4 Statistical modelling of sleep quality data

Two different statistical analyses were performed to assess the quality of sleep of the 12 participants in Roses. First, we analyzed the sleep quality score given by the smartwatch. A linear mixed model was fit to assess the sleep quality score after each activity, including the individual sleep quality score measured before the activity as baseline, activity group as a fixed effect, and session and individual ID as random effects.

Second, we assessed changes between sleep patterns in its phases (light, deep and REM) via multivariate analysis of variance (MANOVA). As the data consisted of the percentage distribution of time spent across the three sleep phases, this conferred on them the special nature of compositional data, i.e. relative data subject to a constant-sum constraint (100%). This prevented the direct use of ordinary MANOVA, so log-ratio transformed data following [40] were applied instead.

## 3 Results

### 3.1 Descriptive statisticsof the study sample

The following table (Table 2) summarizes participants’ initial information (N = 21) and the final population characteristics (N = 16).

The article "Blue prescription: A pilot study of health benefits for oncological patients of a short program of activities involving the sea" was published in 2023. Journal: Heliyon.

**Table 2:** Description on the initially included study population (N = 21) and finally included population (N = 16).

Variable	Initially included population (N = 21)		Finally included population (N = 16)	
	Mean (SD)	Min-Max	Mean (SD)	Min-Max
Age (years)	55 (8.4)	43–71	54 (8.7)	43–71
Household size	3 (0.9)	1–4	3 (1.0)	1–4
Children under 16 years old	0.4 (0.6)	0–2	0.6 (0.6)	0–2
Days/week visit green space	3.8 (2.2)	0–7	3.6 (1.8)	1–7
Days/week visit blue space	4 (2.7)	0–7	3.8 (2.5)	0–7
Days/week intense PA	2 (2.3)	0–7	1.8 (2.1)	0–7
Days/week moderate PA	3.2 (2.4)	0–7	2.6 (2.2)	0–7
Days/week of a 10-min walk	6 (1.6)	2–7	5.9 (1.7)	2–7
	**Freq.**	**Freq. (%)**	**Freq.**	**Freq. (%)**
Gender				
Female	15	71%	14	87,5%
Male	6	29%	2	12,5%
Education				
Did not complete primary	1	5%	1	6%
Completed primary	5	24%	4	25%
Complete secondary	5	24%	4	25%
Complete higher	10	48%	7	44%
Personal finances				
Comfortable	9	43%	8	50%
Intermediate	7	33%	6	37,5%
Some difficulty	5	24%	2	12,5%
Financial struggle	0	0%	0	0%
Home access to open space				
Private garden	6	29%	6	37,5%
Community garden	5	24%	2	12,5%
Balcony/Backyard	4	19%	4	25%
No access to open spaces	1	5%	0	0%
No access but sea views	5	24%	4	25%
Home close to green space				
No	0	0%	0	0%
Yes	21	100%	16	100%
Home close to blue space				
No	2	10%	2	12,5%
Yes	19	90%	14	87,5%

The final study population (N = 16) was made up mostly of women (87.5%), ranging from 43 to 71 years old, living with two other people. Half of participants (50%) felt comfortable in their financial situation, and 69% of them had at least a secondary level education. On average, participants reported visiting green and blue spaces four days a week and performing intense and moderate physical activity two to three days a week.

Five of the participants did not complete all the stages of the study. Three of them reported financial difficulties, which added to the reported health problems and the need to take care of elder relatives of others, which may have been the reasons for abandoning the study.

### 3.2 Mental health

#### 3.2.1 Overall POMS scores

Fig. 3A shows the distribution of the overall POMS scores (combined and by activity group) at pre- and post-activity times. Lower POMS scores are indicative of people with more stable mood profiles. The pre-activity POMS values are generally similar, except for the higher variability observed before the beach activity. A slight overall decrease in POMS scores was observed in the post-activity data, particularly with respect to the control activity and with a more marked decrease after walking and snorkelling.

The article "Blue prescription: A pilot study of health benefits for oncological patients of a short program of activities involving the sea" was published in 2023. Journal: Heliyon.

**Fig. 3:** A) Distribution of overall POMS scores before and after each activity. B) Predicted means of overall POMS scores with 95% confidence intervals from GLMM fit (expressed as rates relative to baseline level).

Among the adjustment variables considered in this analysis, the statistical significance testing suggested that none of them except for “having children under 16” may be relevant for the POMS score. Table 3 shows estimates from final GLMM fits to overall POMS score and POMS scores by category, including activity as fixed effect (and “having children under 16” for model adjustment) and individual ID nested within location as random effect. A marginal statistical significance of the effect of activity on overall POMS scores is indicated (p = 0.04). Table 3 includes predicted means from the model for post-activity overall POMS score by activity category as an explanatory factor of main interest. The means are provided in the original scale and relative to the baseline level for overall comparisons (“***rate***” heading followed by an asymptotic 95% confidence interval for the prediction). Fig. 3B shows the predicted means for overall POMS. Last, Table 3 includes results from post hoc pair-wise comparisons between activities from the GLMM estimates. Although the pair-wise comparisons are not statistically significant, we can observe an overall tendency of decreasing overall POMS scores with an increasing degree of contact with water (or blue space).

**Table 3:** Comparisons between activities of overall POMS scores and split by category.

Outcomes and Variables	Rate (95%CI)	Post hoc comparison	*p*
**Overall POMS score**		Model significance	0.04*
Control	0.98 (0.94–1.03)	Control-Walk	0.37
Walking	0.96 (0.92–1.01)	Control-Beach	0.13
Beach	0.95 (0.90–1.00)	Control-Snorkel	0.07
Snorkel	0.94 (0.89–0.99)	Walk-Beach	0.47
		Walk-Snorkel	0.36
		Beach-Snorkel	0.63
**Tension-anxiety score**		Model significance	0.02*
Control	0.77 (0.65–0.95)	Control-Walk	0.30
Walking	0.70 (0.57–0.86)	Control-Beach	0.02*
Beach	0.60 (0.49–0.74)	Control-Snorkel	0.02*
Snorkel	0.60 (0.48–0.74)	Walk-Beach	0.18
		Walk-Snorkel	0.18
		Beach-Snorkel	0.98
**Fatigue score**		Model significance	0.01*
Control	0.90 (0.55–1.47)	Control-Walk	0.03*
Walking	1.21 (0.74–1.97)	Control-Beach	0.84
Beach	0.87 (0.53–1.41)	Control-Snorkel	0.84
Snorkel	0.85 (0.52–1.38)	Walk-Beach	0.01*
		Walk-Snorkel	0.01*
		Beach-Snorkel	0.84
**Anger-hostility score**		Model significance	0.03*
Control	0.84 (0.62–1.13)	Control-Walk	0.99
Walking	0.84 (0.62–1.12)	Control-Beach	0.03*
Beach	0.53 (0.40–0.70)	Control-Snorkel	0.50
Snorkel	0.72 (0.54–0.98)	Walk-Beach	0.03*
		Walk-Snorkel	0.50
		Beach-Snorkel	0.14
**Depression score**		Model significance	0.86
**Vigour score**		Model significance	0.06
Control	0.97 (0.86–1.10)	Control-Walk	0.24
Walking	1.06 (0.94–1.19)	Control-Beach	0.24
Beach	1.05 (0.93–1.18)	Control-Snorkel	0.04*
Snorkel	1.11 (0.99–1.25)	Walk-Beach	0.84
		Walk-Snorkel	0.39
		Beach-Snorkel	0.34

POMS scores by categories.

The article "Blue prescription: A pilot study of health benefits for oncological patients of a short program of activities involving the sea" was published in 2023. Journal: Heliyon.

Table 3 summarizes the results of the assessment of the significance of the differences in means between activities across the categories of the POMS test. For the Tension-Anxiety score, overall significant differences were concluded between activities (p = 0.02). Although the predicted mean POMS scores are not neatly differentiated between activities, a decreasing trend with the “blue” intensity of the activity is also observed here. In this case, post hoc comparisons show significant differences between snorkel and beach activities with the control activity (p = 0.02).

Irrespective of the result of the statistical significance testing for the fatigue score (p = 0.01), the predicted mean scores and the overlapping associated confidence intervals suggest small effects of the “blue activities” on fatigue. In this case, walking produces somewhat higher scores in comparison to the rest of activities.

Predicted mean scores are again not neatly differentiated across activities for the Anger-Hostility score, but some differences (p = 0.03) are apparent between control and beach activities and between walking and beach activities, with the later activity associated with a somewhat lower mean POMS score.

No statistically significant overall differences in mean depression scores were concluded so no results by activity are reported. Last, a marginally non-significant effect of activity on vigour scores was obtained (p = 0.06). As expected, the predicted mean scores are not neatly differentiated across activities, but an increasing trend with the “blue” intensity of the activity is shown. Post hoc pairwise comparisons only conclude marginally significant differences between the control and snorkelling activities (p = 0.04).

### 3.3 Contribution of activity to SBP, DBP and heart rate measured using a sphygmomanometer

The LMM fit indicated that activity group as main fixed effect appeared not to have a statistically significant association with either the SBP (p = 0.20) or DBP (p = 0.78) variables, which showed similar distributions before and after the activity. The adjustment variables age, weight, height, and usual activity levels (days per week of low, medium and intense activity) were also shown to be non-significant. However, regarding HR (Fig. 4A), values increased prior to doing the “blue” activities, and there appeared to be some patterns in the HR distributions after doing the activity, with tendencies to higher values for HR after walking by the sea and lower values after snorkelling (relative to baseline pre-activity values).

The article "Blue prescription: A pilot study of health benefits for oncological patients of a short program of activities involving the sea" was published in 2023. Journal: Heliyon.

**Fig. 4:** A) Distribution of HR values of the participants before and after each activity. B) Predicted means of post-activity HR expressed as rates relative to baseline level, with 95% confidence intervals from LMM fit.

Formal statistical analysis by LMM concluded a statistically significant effect of activity on HR (p < 0.01). Predicted post-activity means are represented in Fig. 4B, suggesting that, considering baseline pre-activity levels, walking tends to increase HR, while the beach and snorkelling activities show HR values similar to or lower than the control activity.

### 3.4 Contribution of Activities to HR and sleep quality measured using smartwatches

Results on the outcomes obtained by the smartwatches are available in Appendix 2.

## 4 Discussion

To our knowledge, this is the first experimental study on oncological patients to assess both physical and mental health parameters, reporting the health benefits of a short program of different physical activities in a blue space. Our results show that non-motorised activities such swimming, snorkelling and walking along the coast benefit the mental health and well-being of oncology patients, thus providing further evidence of the health benefits of exposure to blue space to the well-being of people with cancer.

We observed that psychological distress in oncological patients with non-active tumours in the remission phase was reduced after taking part in hour-long snorkelling sessions, showing a tendency towards improved mood state (based on POMS scores) with increasing exposure to “blue” activities (i.e. more benefits as the contact with water increased). Thus, our study provides further evidence that exposure to blue spaces contributes to improving human well-being, particularly among people with chronic conditions. Regarding physical health parameters, particularly HR, we observed the same HR reduction as the control after doing the beach and snorkelling activities, while walking activity increased HR. Last, no significant differences were observed in HR measured by smartwatches in any of the different time periods or as regards sleep quality, withno observed changes in sleep scores or sleep stage patterns.

While for the total POMS score we observed a tendency towards improved mood state with increasing exposure to “blue” activities, results showed that different activities lead to different outcomes regarding specific psychological mood parameters. For instance, walking provided worse scores for fatigue, while swimming from the beach caused a reduction in anger-hostility feelings compared with the other activities. Increasing exposure to a blue space also seems to reduce tension-anxiety mood states and increase vigour scores, with snorkelling having the strongest effect.

The article "Blue prescription: A pilot study of health benefits for oncological patients of a short program of activities involving the sea" was published in 2023. Journal: Heliyon.

This correlates with our previous work, where we stated that scuba divers taking regular medication for chronic illness had significantly better POMS vigour scores than the control participants after a short-term exposure to scuba diving [8]. Moreover, our results for mental well-being also concur with the results of six studies assessing the benefits of dragon boat racing involving 67 women with breast cancer, where participants reported enhanced self-confidence, feelings of camaraderie, renewed fitness and health and opportunities to promote awareness of a full and enjoyable life after breast cancer [29,78]; and another study involving 100 women, who had improved results in a health-related quality of life (HRQOL) questionnaire and a reported a decrease in fatigue after a season of dragon boat training [62].

We also observed positive outcomes when comparing HR before and after the activities. The same HR reduction was observed after doing physical activities that involved full contact with the seawater (swimming and snorkelling) as after doing no activity (control), and a tendency to be even lower in the case of snorkelling. This may be in line with an increasingly studied phenomena known as the “diving reflex” [6,7,9,45], where having the face submerged in water contributes to reducing HR as a response to an increased oxygen yield [27]. To this effect, physical activities involving being submerged partially or totally in water, and particularly the face, are suitable even for participants with tachycardias, as this effect may contribute to stabilizing HR [27]. As can be seen, both the beach and snorkelling activities contribute strongly to improving patients’ mental health by reducing tension and improving vigour compared to walking by the coast, while not having the drawback of increasing the participants HR after the training session, which probably contributes to decreased fatigue perceptions.

However, regarding the HR data obtained from the smartwatches, we observed no significant differences in any time period registered or “After”, the time period that correlates with the one-off HR measured with a sphygmomanometer. Despite showing no significant differences in statistical terms, a tendency for HR to be somewhat lower for snorkelling than for the other activities can be seen, which probably reflects the “diving reflex” stated previously [27]. Fig. 5 (Appendix 2) also shows a slight tendency towards HR frequencies before waking up (both the night before exercising and the night after exercising) being slightly lower for all activities compared to the control, and somewhat higher after 30 min of being asleep. This result contrasts with other works, in which an increase in resting heart rate the night after performing very strenuous physical activity has been observed [66,69], and others that have associated 30 min of moderate-high intensity of exercise [46] with lower quality of sleep [17,31]. However, this increment was not detected when participants did 30 min of low level physical activity [46], which correlates with the results obtained in our study. The physical activities proposed in our study should therefore be classified as low demanding when done for 30 min, causing no negative outcomes for oncological patients in terms of their resting heart rate.

The article "Blue prescription: A pilot study of health benefits for oncological patients of a short program of activities involving the sea" was published in 2023. Journal: Heliyon.

Lastly, no significant changes were observed either in the quality of sleep score or the distribution of sleep stages for any of the activities proposed. Previous studies have reported increased total sleep time and deep sleep, and reduced REM sleep, after moderate-high intensity exercise sessions [16], and this was associated with an overall improvement in sleep quality [46]. However, other studies state that these parameters are somewhat difficult to evaluate in sport interventions, as there is a lack of consensus on sleep quality parameter evaluation [71], with sleep quantity in other studies remaining inconclusive, as reported for an 11-week swimming training program in adolescents, which found no significant differences [33]. Nevertheless, even in patients with sleep impairments, most studies reflect slightly significant improved sleep quality, which is mostly self-reported by participants and involves longer training programs [34,85]. However, in a study involving patients with stage IV lung and colorectal cancer on an eight-week training program of a minimum of four days of home-based physical activity, participants self-reported significant improvements in their sleep quality [12]. These results may suggest that when using smartwatches to register changes in sleep patterns, more days of exercise of a greater intensity, or longer training session are required, with the most consistent results on sleep quality obtained with exercise durations of 1 h or more, according to Ref. [16].

Most previous studies have focused on investigating or exploring the benefits for well-being of dragon boat racing among women who have survived breast cancer [5]. Although these studies assess well-being using qualitative in-depth interviews, the positive outcomes in terms of mental health are similar to those reported in our study (McDnonough et al., 2008; [54]. To this effect, while these studies focused only on interviews with women who had done dragon boat racing, we examined different physical activities in a population with no previous experience that was of a similar volume (3–20 persons) and age range (40–75 years) as the dragon boat racing studies. Nevertheless, these findings show a clear benefit for mental health, which must be understood as indissociable with physical health, providing an opportunity to investigate the contribution of doing physical activities in a blue space to both physical and mental health in people recovering from cancer. Therefore, further studies on larger groups of patients need to be undertaken that assess both the physical and mental health benefits of doing maritime recreational activities, and especially those thati nvolve full contact with the seawater, for the purpose of developing health promotion programs to meet the patients’ needs for follow-up post-treatment care and support activities [52].

The article "Blue prescription: A pilot study of health benefits for oncological patients of a short program of activities involving the sea" was published in 2023. Journal: Heliyon.

### 4.1 Strengths and limitations of the study

Despite the novelty of this research, there are several strengths and limitations that must be acknowledged. First, we found no significant results using the data obtained with the smartwatches for either heart rate or sleep quality. However, we believe that these devices provide a unique opportunity to carry out future research, engage patients, and as a means of communication between patients and physicians. As stated in the review by Ref. [64]; smartwatches record data 24/7 and as now affordable devices can be a very useful tool for physicians to gather patient data and more accurately monitor their habits and lifestyle [41,64].

Some studies have shown smartphone application-based physical activity interventions to be effective in promoting physical activity and quality of life among breast cancer survivors, although little research has been conducted on the effectiveness of smartwatches in promoting this population's health [50,58,59]. To this effect, we experienced a general participant acceptance of the devices provided, most of them reporting feeling empowered as they were able to access the data gathered for the study in an understandable way, making them feel they were participating actively both in the study and in their health. However, it must be noted that smartwatches are not as accurate as other HR-monitoring and sleep quality measurement methods [48] and, as seen in our study where “After” time period measurements overlapped between the smartwatches and the sphygmomanometer, differences in results between measurement methods may be reported. Therefore, we encourage further studies to be developed in coordination with health care professionals using smartwatches, but without relying only on this method of measurement and using complementary alternatives such as waist-based HR registering devices or sleep tracking devices to obtain the most accurate and precise results.

The article "Blue prescription: A pilot study of health benefits for oncological patients of a short program of activities involving the sea" was published in 2023. Journal: Heliyon.

Second, although we found mental health benefits related to the degree of exposure to blue spaces when compared to the control group, different controls could be made for other interesting comparisons. An example to this effect would be an additional control group that did short walks in a closed or urban space, or bathed/did snorkelling in a swimming pool [80]. In addition, it would be interesting to compare these groups with subjects doing activities in green spaces (i.e. forest walking guided tours, recreational walks, interactively studying local fauna and flora, etc.), as many studies have reported that these also have beneficial outcomes for mental health [10,11,13]. Last, each participant was their own control prior to taking part in the activities, which on the one hand is positive in terms of avoiding biases when comparing the effects of “blue” activities, but on the other hand is negative since the order in which the activities were carried out could have influenced the results. Therefore, further studies need to be carried out with a higher number of subjects, grouping them but altering the order in which the activities are carried out between groups, and using different controls or comparisons between urban, green and blue spaces.

Third, there were several logistic difficulties derived from managing a group of oncological patients in the context of a pandemic. Several participants were lost from the sample, reporting problems such as financial struggles and timetable incompatibilities between sessions and their jobs. These issues are summarized in Appendix Table 1 and recommendations are also proposed to avoid these problems in future research, for example organizing sessions at different times (e.g. morning and afternoon) to allow participants to schedule the activities depending on their jobs, medical appointments, self-care and care of relatives. These adherence issues must also be considered when implementing future social prescription programs in primary healthcare.

Fourth, despite an overall acceptance on the part of patients regarding the use of the smartwatches, most of them were using these devices for the first time. This issue can mean disturbances to patients’ comfort and the inability to solve problems when the device malfunctions. These issues are covered in Appendix Table 2, along with recommendations to solve the problems detected in this study.

The article "Blue prescription: A pilot study of health benefits for oncological patients of a short program of activities involving the sea" was published in 2023. Journal: Heliyon.

Fifth, regarding gender, we only managed to recruit six males for this study, and only two of them completed all the activities. This bias is not surprising, as studies indicate that men are less likely to take part in cancer support groups than women [35,68,81]. To this effect, a strategic approach should be taken to reduce this gender gap and encourage more men to take part in studies or activities of this type. Primary healthcare professionals play a crucial role in developing a trust-based relationship and engaging male individuals, who are generally more reluctant to this effect.

Sixth, in the present study we only assessed the short-term benefits of three different types of activities in a blue space (i.e. walking, beach and snorkelling). It would be interesting to further explore how long these health benefits continue after the exposure, or how consistently these activities need to be done for sustained and long-term benefits.

Lastly, it must be noted that due to the expected difficulty of recruiting participants that met the study requirements, no power calculations were made and the final sample of this study was limited in size. Moreover, due to several participants in Tossa de Mar abandoning the study, the analyses of the smartwatch data were based only on the Roses data. Therefore, it must be stated that this study is a preliminary investigation. Further studies using the present one as a basis to inform refinements as to the design and methodology are required to confirm the suggested effects and to shed more detailed light on the research question.

### 4.2 Future direction

Community-based interventions, also known as social prescriptions, are gaining popularity as a means of providing non-medical support to patients with chronic conditions, including cancer (Lester et al., 2007; South et al., 2008; [52]. Their purpose is to link patients in primary care with sources of support within the community and to provide general practitioners (GPs) and social workers with a non-medical referral option that can operate alongside existing treatments to improve health and well-being [4]. There is growing scientific evidence that these interventions can lead to positive outcomes, and public health services in some countries, including the UK and Spain, have implemented social prescribing programs to promote health and well-being [4,65].

Green prescriptions, which involve exposure to natural environments through regular walks in a green space (forests, countryside, parks, etc.) or gardening programs [4,36,65,79], have been established as an innovative way to improve physical and mental health [63]; but blue spaces have just recently stepped into this scenario.

The article "Blue prescription: A pilot study of health benefits for oncological patients of a short program of activities involving the sea" was published in 2023. Journal: Heliyon.

The results obtained in this research can serve as a cornerstone to promote further community-based support interventions focused on individuals living beyond cancer, enabling them to engage in a variety of sea activities and services that may reduce the impact of their diagnosis and improve their health and well-being. The proposed intervention in this research was well-received among town councils, primary health care centers, patients’ associations and local stakeholders, who were eager to extend this community-based intervention research to more collectives and other leisure activities in blue spaces. Collaboration between ocean researchers, health professionals, oncology patients and coastal communities can deliver a resilient, sustainable ocean that fosters improvements in public health, which is of paramount importance given the United Nations announcement of the Decade of Ocean Science for Sustainable Development from 2021 to 2030 [18]. Therefore, further research, in coordination with other health professionals and local collectives, is encouraged to determine the real impact of leisure activities in blue spaces on social prescribing for patients with health needs and chronic conditions.

## 5 Conclusions

In the present study, a gradient of positive results for human mental health can be observed. Beach and snorkelling activities contribute to reducing tension and anger and improving the vigour mood state of oncological patients with no significant changes in heart rate or sleep quality. Therefore, these activities may promote relaxation and can be classified as low demanding, making them suitable for patients with similar characteristics to those enrolled in the study.

Further studies are needed to evaluate the potential benefits of activities related to blue spaces on the mental health and well-being of oncological patients in the short, medium, and long term. Health promotion programs such as blue prescriptions should be implemented to help patients access blue spaces, activities, services, and support in their community.

## Author contribution statement

Carreño, Arnau conceived and designed the experiments; performed the experiments; analyzed and interpreted the data; contributed reagents, materials, analysis tools or data; wrote the paper.

Fontdecaba, Eva; conceived and designed the experiments; performed the experiments.

Izquierdo, Angel conceived and designed the experiments.

Enciso, Olga conceived and designed the experiments; performed the experiments.

Daunis-i-Estadella, Pepus analyzed and interpreted the data; contributed reagents, materials, analysis tools or data; wrote the paper.

The article "Blue prescription: A pilot study of health benefits for oncological patients of a short program of activities involving the sea" was published in 2023. Journal: Heliyon.

Mateu-Figueras, Gloria analyzed and interpreted the data; contributed reagents, materials, analysis tools or data; wrote the paper.

Palarea-Albaladejo, Javier analyzed and interpreted the data; contributed reagents, materials, analysis tools or data; wrote the paper.

Gascon, Mireia analyzed and interpreted the data; contributed reagents, materials, analysis tools or data; wrote the paper.

Vendrell, Cristina conceived and designed the experiments.

Lloveras, Montserrat conceived and designed the experiments.

San, Joan conceived and designed the experiments.

Gómez, Sílvia conceived and designed the experiments; performed the experiments.

Minuto, Stefania performed the experiments.

Lloret, Josep conceived and designed the experiments; performed the experiments; contributed reagents, materials, analysis tools or data.

## Data availability statement

The data that has been used is confidential.

## Declaration of competing interest

The authors declare that they have no known competing financial interests or personal relationships that could have appeared to influence the work reported in this paper.

## Figures and Tables

**Fig. 5:** Distribution of standardized HR values for each activity and time of measurement. Dashed line indicates no difference with baseline mean HR in the control session.

**Fig. 6:** Distribution of sleep quality scores by activity.

**Fig. 7:** Distribution of percentages of the different sleep stages analyzed (Light, Deep and REM) for each activity. A) Night before the activity; B) Night after the activity.

**Appendix Table 1:** 

Issue	Problematic	Solution
Recruiting participants	Several potential candidates for this study did not agree to take part for different reasons, including insecurity regarding swimming, the study requiring too much engagement, not wanting to join a group with other people, etc.	Here the physician is crucial in terms of engaging the patient and conveying a sense of security and willingness to participate. Close bonds between primary health care professionals and patients are required to promote the latter's participation.
Participants follow-up	Out of 21 participants in this study, nine failed to follow all the sessions programmed. It is consistently difficult to coordinate a group of participants to be available on certain days and times: work, self-care, care of other relatives, other appointments, etc. Moreover, given that the participants in the study were patients in a recovery phase from cancer, their situation was particularly irregular in terms of medical visits, illnesses and self-care. Additionally, the recent Covid 19 pandemic also meant that we had to adjust our study in line with national constraints, for example not being able to be in a group of more than four people.	
● Health issues	One participant was lost due to reported health problems that prevented her from participating in the swimming and snorkelling sessions.	We encouraged the participant to rejoin the sessions as soon as she felt she could again take part. New sessions were organized for the participants that could not attend.
● Working issues	Six participants were lost due to job issues. When performing a study on a coastal population, the fact that most inhabitants do extended working hours during the tourist season, in this case in summer, must be taken into account. When this issue is combined with doing sea activities which, in the case of these patients, must be when the climate allows (i.e. comfortable air and water temperatures, sea conditions, etc.), these two factors overlap.	We organized different sessions at different times (e.g. morning and afternoon) to allow participants to schedule the activities according to their jobs and other appointments. For example, two sessions were organized on the same day, one in the morning and one in the afternoon; or we repeated the sessions for those who were not able to attend.
● Covid-19	Two participants were lost due to Covid-19 affecting relatives, meaning they could not attend the programmed sessions.	Unfortunately, this is not an issue that can be avoided. We encouraged the affected participants to take part once again when their relatives' condition improved.

The article "Blue prescription: A pilot study of health benefits for oncological patients of a short program of activities involving the sea" was published in 2023. Journal: Heliyon.

**Appendix table 2:** 

Smartwatches		
-Accuracy of monitoring variables	The accuracy of smartwatches in measuring heart rate varies, and none are as accurate as an electrode-containing chest monitor, which approaches the accuracy of an ECG [1]. The accuracy of wrist-based devices can also be affected by factors such as body temperature, hemoglobin levels, skin status, and blood pressure [1,5].	Acquiring better wrist-based devices or combining them with bellyband HR measuring devices would help to lower the bias that smartwatches are subject to.
-Disturbances related to wearing smartwatches	Monitoring both heart rate and quality of sleep implies wearing the smartwatch 24/7, even in situations where the participant may be not used to it, such as wearing the device while sleeping. Almost half the participants complained about the watches being uncomfortable for sleeping or doing their everyday tasks during the first week of the study. One participant also reported an allergy, developing a skin rash on the wrist where the device was worn.	Strategies were adopted to allow participants that reported discomfort to remove the device during the day or at night in between groups of activities. Since the allergy was reported in the interval between the walking and control sessions, the device was removed until the allergy disappeared. No further allergy episodes were reported.
-Not activating the device while performing the activities	Although a training session was held prior to the start of the study where it was explained to participants how to use and charge their devices, some of them experienced difficulties using them. Although we tried to make sure that every device was registering the training session, on very few occasions a participant's device was not activated.	It is advisable to remind participants to turn on their devices and always ensure that all the smartwatches are activated before starting the activity.
-Device malfunctioning	The devices malfunctioned several times, although we do not know if this was a device error or due a participant tampering with the watch, so the HR of some patients stopped being recording on several occasions. Although we always had each patient's smartwatch register to hand and we were able to resolve errors as soon as they were detected, a couple of incidents did remain undetected, leading to a loss of data about HR and sleep quality (dependent on the HR monitoring function being activated).	We strongly recommend reviewing the smartwatches' recording history every day and resolve problems detected due to malfunctioning as soon as possible.
-Removal of the devices	Cases of the participant removing the smartwatch without informing the research team occurred. Despite most of the cases being rapidly detected and the participants redressing the problem, in one case the participant did not follow the research team's repeatedly given instructions and wore the device only during the training sessions. Therefore, the data obtained from this participant is scarce.	We strongly recommend revising smartwatch's’ recording history every day and assure that all the devices are recording all the parameters.

The article "Blue prescription: A pilot study of health benefits for oncological patients of a short program of activities involving the sea" was published in 2023. Journal: Heliyon.

## APPENDIX 1 Questionnaires

Background questionnaires were only completed once by the participants and included the following information: i) Individual characteristics [e.g. gender (i.e. female, male); age (i.e. years of age); owning a dog (yes, no); having access to an open space at home (private garden, community garden, private space to open air but not a garden, no access but views of a natural space, no access and no views); number of people living with them (i.e. number); children under 16 living with them (i.e. number); educational level (incomplete primary education, completed primary education, completed secondary education, completed higher education); purchasing power (significant financial difficulties, with certain financial difficulties, neither living comfortably nor having financial difficulties, living comfortably, does not know/does not want to answer); having a green space within 10–15 min of their residence (yes, no); frequency of visits to the green space (i.e. times/day; times/week); having a blue space within 10–15 min of their residence (yes, no); frequency of visits to the green space (i.e. times/day; times/week)]; and ii) physical activity and health [e.g. number of times per week doing intense physical activity (i.e. weightlifting, digging, aerobic exercise, etc.) (1–7); number of times per week doing moderate physical activity (walking not included) (i.e. light weightlifting, riding a bicycle at a medium speed, etc.) (1–7); number of days per week walking for at least 10 min (1–7); and regular medication intake (yes, no)]. Medication intake was defined as participants who took medication to treat chronic physical or psychiatric illnesses. Medication use included estrogen modulators, testosterone supplements, fluoxetine and mild analgesics.

All participants in the study were asked to answer several questionnaires just before and after taking part in their respective activity sessions (approximately 1 h of difference between questionnaires).

The questionnaires before starting the cluster of activities were only distributed before the first session of each activity and included the following information: i) perception of health [e.g. own perception of their health (1–5); happiness the previous day (1−10); anxiety the previous day (1−10); satisfaction with life (1−10); things in their life of worth (1−10)]; and ii) physical activity [e.g. visiting blue spaces in the previous 4 weeks (i.e. times per week); number of times the previous week doing intense physical activity (i.e. weightlifting, digging, aerobic exercise, etc.) (0–7); number of times the previous week doing moderate physical activity (walking not included) (i.e. light weightlifting, riding a bicycle at a medium speed, etc.) (0–7); number of days the previous week walking for at least 10 min (0–7)].

The questionnaires before the sessions included the following information: i) How they felt the previous day and how they had slept [e.g. easy to sleep the previous night (1–5); disturbed sleep the previous night (1–5); woke up earlier than usual (1–5); overall quality of sleep (1–5); and number of hours of sleep]; and ii) POMS section.

The questionnaires after the session included the following information: i) Activity (control, walking, beach or snorkelling) session characteristics [e.g. uncomfortable because of the noise (1–5); uncomfortable because of people (1–5); uncomfortable because of pollution (1–5); uncomfortable because of fishing gear (1–5); happiness while doing the activity (1–5); active while doing the activity (1–5); feeling safe while doing the activity (1–5)]; and ii) POMS section.

The article "Blue prescription: A pilot study of health benefits for oncological patients of a short program of activities involving the sea" was published in 2023. Journal: Heliyon.

The questionnaires after completing the cluster of activities were only distributed after the last session of each activity and included the following information: i) perception of health [e.g. own perception of their health (1–5); happiness the previous day (1−10); anxiety the previous day (1−10); satisfaction with life (1−10); things in their life of worth (1−10); waking up fresh and well rested during the activity week (1–6); feeling motivated with life during the activity week (1–6)] ii) physical activity [e.g. visiting blue spaces during the week of activity (i.e. times per week); number of times during the week of activity doing intense physical activity (i.e. weightlifting, digging, aerobic exercise, etc.) (0–7); number of times during the week of activity doing moderate physical activity (walking not included) (i.e. light weightlifting, riding a bicycle at a medium speed, etc.) (0–7); number of days during the week of activity walking for at least 10 min (0–7)].
